The article "The Characteristics of Fear of Recurrence and the Effect of Cognitive-Behavioral Stress Management Intervention in Patients after Radiofrequency Ablation of Atrial Fibrillation" was retracted in 2023. Reasons: unreliable results or conclusions; lack of ethics approval or compliance; concerns about the data; concerns about the peer review.

# The Characteristics of Fear of Recurrence and the Effect of Cognitive-Behavioral Stress Management Intervention in Patients after Radiofrequency Ablation of Atrial Fibrillation

**DOI:** 10.1155/2022/6916302

**Published:** 2022-07-20

**Authors:** Juan Chen, Lu Qian, Cuilian Chen, Xiaoling Wang

**Affiliations:** Department of Cardiology, The First Affiliated Hospital of Soochow University, Suzhou 215031, China

## Abstract

The aim of this study was to grasp the current situation of fear of recurrence in patients after radiofrequency ablation of atrial fibrillation and to explore the application effect of cognitive-behavioral stress management in patients with fear of recurrence after radiofrequency ablation of atrial fibrillation. From July 2020 to July 2021, 150 patients with fear of recurrence of atrial fibrillation after radiofrequency ablation in our hospital were divided into a control group and an intervention group, with 75 cases in each group. Both groups received conventional nursing methods, and the intervention group received 8 weeks of cognitive-behavioral stress management. Before the intervention and after the intervention, the general situation questionnaire, the Chinese version of the Fear Disease Progression Simplified Scale (FoP-Q-SF), the Perceived Stress Scale (CPSS), and the Positive Psychological Capital Questionnaire (PPQ) were used for evaluation. Before the intervention, there were no significant differences in general data, degree of fear of recurrence, stress perception, and psychological capital scores between the two groups (*P* > 0.05). After 8 weeks of cognitive-behavioral stress management intervention, the fear recurrence, the total score of stress perception, and the scores of each dimension in the intervention group were significantly lower than those in the control group, and the psychological capital score was significantly higher than that in the control group, with statistically significant differences (*P* < 0.05). Cognitive-behavioral stress management method can significantly reduce the fear of recurrence and stress level of patients after radiofrequency ablation of atrial fibrillation, and improve their psychological capital level.

## 1. Introduction

Atrial fibrillation is a chronic heart disease with chronic arrhythmia as the main manifestation, and its prevalence increases with age [1]. The current study shows that the recurrence rate of nonelderly patients within 1 year after radiofrequency ablation (RFA) is 7.50%, and the recurrence rate of elderly patients is as high as 17.14% [2], which greatly increases the psychological burden of patients and leads to fear of cancer recurrence (FCR) occurs after surgery. Long-term FCR can reduce the quality of life of patients and induce psychological distress and maladaptive behaviors, and appropriate intervention is urgently needed. Cognitive-behavioral stress management is a psychotherapeutic approach that combines cognitive-behavioral theory and relaxation techniques to achieve effective psychological intervention by increasing awareness of stressors and indicators of stress [3]. Mainly through the teaching of cognitive-behavioral stress management methods in the form of preaching, combined with practical exercises of relaxation training [4], there have been reports in China that cognitive-behavioral stress management has a special effect on fear recurrence in young breast cancer patients after surgery [5]. This research intends to quest the feasibility and application effect of CBSM in patients with FCR after RFA of atrial fibrillation and to provide a reference for relieving patients' FCR and constructing precise intervention for patients after RFA of atrial fibrillation. The report is as follows.

The article "The Characteristics of Fear of Recurrence and the Effect of Cognitive-Behavioral Stress Management Intervention in Patients after Radiofrequency Ablation of Atrial Fibrillation" was retracted in 2023. Reasons: unreliable results or conclusions; lack of ethics approval or compliance; concerns about the data; concerns about the peer review.

## 2. Objects and Methods

### 2.1. Survey Objects

From July 2020 to July 2021, 150 patients with atrial fibrillation after RFA in the Department of Cardiovascular Medicine of our hospital were selected as the research subjects. In the light of the random number table, 150 patients were separated into the intervention group and the control group, with 75 patients in each group. Inclusion criteria were as follows: (1) patients with nonvalvular paroxysmal atrial fibrillation aged 18 to 75 years old, and unwilling to adhere to oral anticoagulants for a long time; (2) first time performing cardiac radiofrequency ablation and signed the informed consent form before surgery; (3) fear of recurrence: FoP-Q-SF score ≥ 34 points. Exclusion criteria were as follows: (1) acute and chronic infections; (2) severe valvular stenosis or heart failure; (3) hyperthyroidism; (4) patients with psychiatric disorders, communication barriers, and unable to cooperate with filling out the scale; (5) patients who have undergone cardiac surgery within 3 months before surgery; (6) patients with liver and kidney insufficiency; (7) patients with malignant tumors; and (8) patients with blood diseases and coagulation disorders.

### 2.2. Methods

The control group was offered routine treatment and nursing education including preoperative guidance, psychological care, medication guidance, and dietary guidance and issued the “Health Education Manual for Patients After RFA of Atrial Fibrillation.” At the time of discharge, the doctor will formulate a postdischarge treatment plan, and the responsible nurse will provide rehabilitation guidance to the patient, inform the patient of the regular outpatient review time, and provide rehabilitation guidance and support during the outpatient review.

The article "The Characteristics of Fear of Recurrence and the Effect of Cognitive-Behavioral Stress Management Intervention in Patients after Radiofrequency Ablation of Atrial Fibrillation" was retracted in 2023. Reasons: unreliable results or conclusions; lack of ethics approval or compliance; concerns about the data; concerns about the peer review.

On the basis of the control group, an intervention group was established. The intervention group consisted of 7 members: one chief physician and one deputy chief physician of the Department of Cardiology, responsible for formulating postoperative treatment plans and controlling risks; 5 nurses with 2 years of working experience in cardiovascular medicine, responsible for postoperative teaching, evaluation and guidance and follow-up work of patients, the abovementioned personnel are all qualified for intervention training. The intervention group implemented CBSM intervention mainly by group intervention and supplemented by “one-to-one.” The group consists of 3–5 people, 150 min/time/week, of which 120 min is stress management, 30 min is relaxation training, and the intervention is continued for 8 weeks. The specific methods are as follows.

#### 2.2.1. Group Intervention

(1) Cognitive reconstruction: intervention in the form of lectures, combined with self-made PPT and videos, to introduce the basic knowledge of the disease, factors affecting recurrence and prognosis, so that patients can clearly understand the relationship between the fear of recurrence and the source of stress after surgery, and both effects, negative effects. At the same time, through classroom questions, guide group members to share their anxiety, source of fear, stress status, and under the guidance of nurses, how to overcome these negative emotions and create a good atmosphere for patients. (2) Behavioral intervention: as the patients lie down for a long time after the operation, the nursing staff should instruct the patients and their accompanying staff on how to solve the problem of two bowel movements, to avoid the resulting anxiety. At the same time, the thigh root of the patient is tightly bandaged after surgery, and pain and discomfort are common. Instruct the patient on how to turn over and move the body, and moderately loosen the bandage if necessary. To ease the patient's discomfort, you can also play relaxing music to ease the patient's tension. (3) Social support training: organize patients to communicate with each other, invite patients with a good mental state of postoperative recurrence, share the experience of how to maintain a good state of mind, and transfer positive energy to each other. At the same time, the nursing staff also needs to fully understand the psychological needs of the patients, and ask the family members to give more care, comfort, understanding, and encouragement, to encourage the patients to face the pain bravely, which will help reduce the fear of postoperative recurrence. (4) Relaxation training: the trained and qualified nurses carry out progressive relaxation training, instructing patients to clench their fists to experience the feeling of tension when inhaling for a few seconds, and slowly relax their fists to experience the feeling of relaxation when exhaling for a few seconds. Then contract and relax your hands, arms, face, neck, shoulders, and other muscle groups in turn, 20–30 min/time, to ensure that each movement is in place. According to the patient's hobby, play relaxing music and comedy movies, and transfer and relieve the patient's negative emotions.

The article "The Characteristics of Fear of Recurrence and the Effect of Cognitive-Behavioral Stress Management Intervention in Patients after Radiofrequency Ablation of Atrial Fibrillation" was retracted in 2023. Reasons: unreliable results or conclusions; lack of ethics approval or compliance; concerns about the data; concerns about the peer review.

#### 2.2.2. Individual Intervention

Intervention in the form of “one-on-one,” whether it is online or offline platforms, conduct a psychological assessment of patients, timely relieve existing negative emotions, answer patients' questions in detail, encourage and support, monitor patients' daily activities, and give routine behavioral intervention, social support training, and relaxation training.

### 2.3. Evaluation Tools and Observation Indicators

The general information questionnaire includes 13 items, including age, BMI, gender, education level, employment status, marital status, the monthly average income of the family, payment method of medical expenses, place of residence, disease understanding, type of atrial fibrillation, concurrent chronic diseases, and main caregivers.

(1) The FoP-Q-SF scale adopts the Chinese version of the fear of progression questionnaire-short form (Fear of progression questionnaire-short form, FoP-Q-SF), which has been localized and revised by domestic scholars Wu [6] and others to investigate patients. The simplified scale includes 2 dimensions of physical health and social family function, each dimension has 6 items, altogether 12 items. According to the Likert 5-level scoring method, each item has distributed a score of 1–5 from “strongly disagree” to “strongly agree,” with a total score of 12 to 60. The higher the score, the higher the patient's fear level, and the whole score ≥ 34. Scores indicate that patients have fear of recurrence after radiofrequency ablation. (2) Perceived Stress Scale [7] (CPSS) mainly includes 2 dimensions of loss of control and tension, with a total of 14 items. Scoring standard: Likert 5-level scoring method, with a score of 0–56, the higher the score, the greater the pressure on the patient. Evaluation criteria: the total score of ≤ 28 points indicate normal, 29–42 points indicate greater stress, and ≥ 43 points indicate excessive stress. (3) The Positive Psychological Capital Questionnaire (PPQ) adopts the PPQ compiled by Zhang [8]. The questionnaire includes four dimensions (self-efficacy, hope, resilience, and optimism) and a total of 36 items (there are 10 questions in population and sociological factors, and 26 questions in four dimensions), and each factor of the four dimensions is from completely inconsistent to completely consistent, using seven-level scoring, and the higher the score, the higher the level of positive psychological capital of the individual.

The article "The Characteristics of Fear of Recurrence and the Effect of Cognitive-Behavioral Stress Management Intervention in Patients after Radiofrequency Ablation of Atrial Fibrillation" was retracted in 2023. Reasons: unreliable results or conclusions; lack of ethics approval or compliance; concerns about the data; concerns about the peer review.

## 3. Methods of Data Collection

After the patients were enrolled and the 8-week intervention was completed, the scales were distributed uniformly by two nurses, and the patients completed them independently. The questionnaire was completed and collected on the spot. A total of 150 questionnaires were distributed in this study, and 7 questionnaires were not filled out properly, 143 valid questionnaires were recovered, and the effective recovery rate was 95.33%.

### 3.1. Quality Control

When designing the research scheme, this study conducted the scheme design by consulting a lot of relevant literature and cooperating with doctors and nurses with rich undergraduate experience to ensure the feasibility of the scheme. Before filling out the questionnaire, the patient's condition should be fully evaluated, and it can be carried out only after the condition is good and the patient and family members agree. During the process of filling in the questionnaire, due to differences in the cognition of different patients, the researcher should patiently guide the patients to fill in the questionnaires in a standardized manner.

### 3.2. Statistical Methods

SPSS 23.0 statistical software was used for data analysis. Normally distributed measurement data is expressed as mean ± standard deviation ($\bar{x}$ ± *s*), comparison between two groups is by *t*-test, count data is described by frequency and percentage, and comparison between groups is by *χ*2 test, *P* < 0.05 is considered statistically significant difference study meaning.

## 4. Results

### 4.1. Comparison of General Data

Comparison of general data of patients after RFA of atrial fibrillation between the two groups the age, BMI, gender, education level, employment status, marital status, the monthly average income of the family, payment method of medical expenses, place of residence, degree of understanding of the disease, type of atrial fibrillation, concurrent chronic diseases, there were no important differences in general data of the primary caregiver (*P* > 0.05), and they were comparable, as indicated in Table 1.

### 4.2. Comparison of Total FCR Scores and Scores of Physical Health and Social Family in Two Groups of Patients with Atrial Fibrillation after RFA before and after Intervention

The total FCR score of the two groups of patients before the intervention was (39.90 ± 5.08) points, and the total FCR score of the two groups of patients after the intervention was (33.82 ± 2.86) points, and the difference was statistically significant (*P* < 0.05). Before the intervention, there was no significant difference in the physical health score, social family score, and total FCR score between the two groups (*P* > 0.05); after the intervention, the FCR total score and dimension score of the two groups were statistically significant (*P* < 0.05), as indicated in Table 2.

The article "The Characteristics of Fear of Recurrence and the Effect of Cognitive-Behavioral Stress Management Intervention in Patients after Radiofrequency Ablation of Atrial Fibrillation" was retracted in 2023. Reasons: unreliable results or conclusions; lack of ethics approval or compliance; concerns about the data; concerns about the peer review.

### 4.3. Comparison of the Total Score of Perceived Stress and the Two Dimensions of Tension and Loss of Control in Patients with Atrial Fibrillation after RFA before and after Intervention

Before the intervention, there was no significant difference in the overall scores of tension, loss of control, and CPSS between the two groups (*P* > 0.05); statistical significance (*P* < 0.05), as indicated in Table 3.

### 4.4. Comparison of Total Resilience Score, Self-Efficacy, Hope, Resilience, and Optimism between Two Groups of Patients with Atrial Fibrillation after RFA before and after Intervention

Before the intervention, there was no significant difference in the overall PPQ scores of self-efficacy, hope, resilience, and optimism between the two groups (*P* > 0.05), as shown in Table 4 and Table 5.

### 4.5. Comparison of FCR Total Score, CPSS Total Score, and PPQ Total Score before and after RFA Intervention in the Two Groups of Patients with Atrial Fibrillation after RFA

Compared with before the intervention, the total scores of FCR and CPSS in the two groups were significantly decreased, and the total scores of PPQ were significantly increased after the intervention, indicating that the control group and the intervention group after the intervention could reduce the fear of recurrence and the risk of atrial fibrillation in patients after RFA. The stress level was beneficial to improve their psychological capital level, but the intervention effect of the CBSM method was more significant, as shown in Figures 1–3.

## 5. Discussion

RFA is an important treatment for paroxysmal atrial fibrillation and persistent atrial fibrillation unresponsive to medical therapy, with a recurrence rate of up to 30–45% after the first RFA [9]. Based on this, patients with atrial fibrillation after RFA often suffer from the double pressure of disease recurrence and treatment costs, resulting in increased psychological burden and negative emotions such as anxiety and fear. Current studies have confirmed that anxiety after cancer surgery is significantly correlated with fear of recurrence [10]. Liu [11] found that among patients with atrial fibrillation who received radiofrequency ablation, 38.50% of the patients had postoperative anxiety symptoms, and long-term anxiety would lead to FCR. At the same time, the appearance of FCR will aggravate the patient's anxiety, depression, and avoidance symptoms, form a vicious circle, and seriously affect the patient's quality of life. Therefore, for patients after RFA, in addition to certain drug treatments, we must also pay attention to the patient's psychological state. Clinical medical workers and their families should carry out active and effective psychological interventions for patients to reduce the risk of postoperative arrhythmia recurrence.

The article "The Characteristics of Fear of Recurrence and the Effect of Cognitive-Behavioral Stress Management Intervention in Patients after Radiofrequency Ablation of Atrial Fibrillation" was retracted in 2023. Reasons: unreliable results or conclusions; lack of ethics approval or compliance; concerns about the data; concerns about the peer review.

CBSM is a reasonable method to correctly understand stress. It is mainly based on the patient's fear, and guides patients to correctly understand the source of stress and fear, and master the CBSM method, thereby reducing the FCR level of patients with atrial fibrillation after RFA. Russell DC [12] and others have reported that CBSM intervention reduces anxiety, anger, and perceived stress levels. Numerous data demonstrate that CBSM interventions are effective in improving disease resilience in a variety of populations with life-threatening and chronic diseases, including breast cancer [13].

Psychological capital belongs to the category of positive psychology and plays a good mediating role in the disease pressure and quality of life faced by patients. A high level of psychological capital is beneficial for people to avoid disease stress injury and reduce self-perceived burden [14]. Sun H [15] et al reported that the higher the psychological capital, the lower the fear of disease progression. Through effective health coaching and establishing healthy behaviors in patients, anxiety, and depression in cancer patients can be alleviated and their quality of life can be significantly improved. Effective health education can lead to a high fear of worsening the condition.

The total score of FCR before intervention in the two groups of patients after RFA for atrial fibrillation involved in this study was (39.90 ± 5.08), which was at a moderate level, higher than the total score of FCR by Deng [5] et al. (35.44 ± 4.23), suggesting that RFA for atrial fibrillation The level of FCR in postoperative patients is higher than that in young breast cancer patients, and the reason may be related to the influencing factors of FCR. The results of this study showed that there was no significant difference in FCR levels between the control group and the intervention group before the intervention. However, 8 weeks of CBSM intervention in the intervention group could effectively reduce the FCR level of patients with atrial fibrillation after RFA. The total score of CPSS before intervention in the control group was (34.03 ± 5.96), and the total score in the intervention group was (35.69 ± 6.66), and the difference was not statistically significant. However, after the intervention, the total CPSS scores of the two groups were statistically significant. The levels of self-efficacy, hope, resilience, and optimism in the intervention group were higher than those in the control group, indicating that the use of CBSM intervention can effectively improve the psychological capital level of patients. After RFA for atrial fibrillation, it is helpful for patients to overcome the negative psychology of atrial fibrillation. The reason for the analysis may be that after cognitive reconstruction in the intervention group, the relationship between the fear of postoperative recurrence and the source of stress and the negative effects of the two were clarified, and the patients were encouraged to work hard to overcome their negative psychology. Intervention methods are used to relieve postoperative discomfort symptoms of patients, and patients are guided to apply relaxation therapy to fully relax their mind and body, to effectively relieve stress and help patients overcome FCR. Based on the above research results, it is recommended that nurses pay attention to the perceived stress of patients with atrial fibrillation after RFA, encourage patients to deal with negative emotions with a peaceful mind, and prevent patients from falling into blind psychological distress and extreme stress reactions, thereby reducing their perceived stress [16].

The article "The Characteristics of Fear of Recurrence and the Effect of Cognitive-Behavioral Stress Management Intervention in Patients after Radiofrequency Ablation of Atrial Fibrillation" was retracted in 2023. Reasons: unreliable results or conclusions; lack of ethics approval or compliance; concerns about the data; concerns about the peer review.

The disadvantage of this study is that it only investigated patients with atrial fibrillation after RFA in our hospital, the sample size is small, and the sample of this study is not representative enough. Secondly, this study only explores the impact of CBSM on the psychological level and does not consider whether its health behavior has improved, as well as the patients' real experience and cognition of the disease.

## Figures and Tables

**Figure 1:** Comparison of total FCR scores before and after RFA intervention in two groups of patients with atrial fibrillation.

**Figure 2:** Comparison of total CPSS scores before and after intervention in two groups of patients with atrial fibrillation after RFA.

**Figure 3:** Comparison of total PPQ scores before and after RFA intervention in two groups of patients with atrial fibrillation.

**Table 1:** Comparison of general data of patients after RFA of atrial fibrillation between the two groups (n (%)).

Factors	Control group (*n* = 75)	Intervention group (*n* = 75)	*χ * ^2^/*t*	*P*
Age (years)	48.08 ± 14.54	48.25 ± 17.23	0.067	0.947
BMI (kg/m)^2^	21.73 ± 1.95	21.68 ± 1.91	0.169	0.866
Gender			0.107	0.744
Male	37 (49.33)	39 (52.00)		
Female	38 (50.67)	36 (48.00)		
Educational level			2.162	0.142
Junior high school and below	34 (45.33)	43 (57.33)		
High school and above	41 (54.67)	32 (42.67)		
Employment status			1.714	0.190
Not employed	44 (58.67)	36 (48.00)		
Employed	31 (41.33)	39 (52.00)		
Marital status			0.855	0.836
Married	28 (37.33)	25 (33.33)		
Unmarried	27 (36.00)	29 (38.67)		
Divorced	10 (13.33)	13 (17.33)		
Widowed	10 (13.33)	8 (10.67)		
The monthly average income of the family (yuan)			0.427	0.514
<3500	36 (48.00)	40 (53.33)		
≥3500	39 (52.00)	35 (46.67)		
Payment method			0.698	0.403
Medical insurance	43 (57.33)	48 (64.00)		
At own expense	32 (42.67)	27 (36.00)		
Place of residence			2.679	0.102
City	45 (60.00)	35 (46.67)		
Rural	30 (40.00)	40 (53.33)		
Disease awareness			0.252	0.882
Know very well	31 (41.33)	28 (37.33)		
Generally	30 (40.00)	32 (42.67)		
Don't understand	14 (18.67)	15 (20.00)		
Type of atrial fibrillation			0.457	0.796
Paroxysmal	29 (38.67)	27 (26.67)		
Persistent	31 (41.33)	35 (46.67)		
Permanent	15 (20.00)	13 (17.33)		
Coexisting chronic diseases			1.000	0.317
Yes	42(56.00)	48 (64.00)		
No	33(44.00)	27 (36.00)		
Primary caregiver			2.008	0.366
Spouse	34 (45.33)	26 (34.67)		
Children	30 (40.00)	38 (50.67)		
Others	11 (14.67)	11 (14.67)		

The article "The Characteristics of Fear of Recurrence and the Effect of Cognitive-Behavioral Stress Management Intervention in Patients after Radiofrequency Ablation of Atrial Fibrillation" was retracted in 2023. Reasons: unreliable results or conclusions; lack of ethics approval or compliance; concerns about the data; concerns about the peer review.

**Table 2:** Comparison of total FCR scores and scores of physical health and social family in the two groups of patients with atrial fibrillation after RFA before and after intervention ($\bar{\text{x}}$ ± *s*).

Group	Number of cases	FCR total		Physical health		Social family	
		Before meddling	After meddling	Before meddling	After meddling	Before meddling	After meddling
Control group	75 cases	38.89 ± 6.33	27.33 ± 3.92	18.25 ± 3.99	13.41 ± 2.61	20.64 ± 4.67	13.92 ± 2.41
Intervention group	75 cases	38.99 ± 5.81	24.40 ± 2.72	18.00 ± 4.00	12.13 ± 2.04	19.99 ± 4.43	12.27 ± 2.05
*T*	—	0.913	5.327	0.388	3.349	0.879	4.527
*P*	—	0.363	< 0.001	0.698	0.001	0.381	< 0.001

**Table 3:** Comparison of the total score of perceived stress and the two dimensions of tension and loss of control in patients with atrial fibrillation after RFA before and after intervention ($\bar{\text{x}}$ ± *s*).

Group	Number of cases	Total CPSS score		Nervous feeling		Feeling out of control	
		Before meddling	After meddling	Before meddling	After meddling	Before meddling	After meddling
Control group	75 cases	34.03 ± 5.96	26.18 ± 2.70	16.50 ± 4.14	13.16 ± 2.06	17.53 ± 4.18	13.01 ± 2.16
Intervention group	75 cases	35.69 ± 6.66	22.71 ± 2.20	17.57 ± 4.65	12.05 ± 2.33	18.12 ± 4.49	12.39 ± 1.77
*t*	—	−1.609	8.594	−1.489	3.075	−0.835	1.936
*P*	—	0.110	<0.001	0.139	0.003	0.405	0.055

The article "The Characteristics of Fear of Recurrence and the Effect of Cognitive-Behavioral Stress Management Intervention in Patients after Radiofrequency Ablation of Atrial Fibrillation" was retracted in 2023. Reasons: unreliable results or conclusions; lack of ethics approval or compliance; concerns about the data; concerns about the peer review.

**Table 4:** Comparison of total elasticity score, self-efficacy, and hope score before and after intervention in RFA patients ($\bar{\text{x}}$ ± *s*).

Group	Number of cases	Total PPQ score		Self-efficacy		Hope	
		Before meddling	After meddling	Before meddling	After meddling	Before meddling	After meddling
Control group	75 cases	111.51 ± 5.02	122.00 ± 6.77	29.69 ± 3.04	30.80 ± 2.54	27.24 ± 2.70	29.95 ± 3.01
Intervention group	75 cases	110.48 ± 4.69	134.35 ± 6.88	29.35 ± 2.83	33.88 ± 2.82	26.92 ± 2.36	32.05 ± 3.37
*t*	—	1.295	−11.076	0.723	−7.028	0.773	−4.034
*P*	—	0.197	< 0.001	0.471	< 0.001	0.441	< 0.001

**Table 5:** Comparison of resilience and optimism dimension scores in patients with atrial fibrillation after RFA before and after intervention ($\bar{\text{x}}$ ± *s*).

Group	Number of cases	Resilience		Optimism	
		Before meddling	After meddling	Before meddling	After meddling
Control group	75 cases	26.44 ± 2.06	30.80 ± 3.41	28.13 ± 2.73	30.45 ± 3.59
Intervention group	75 cases	26.24 ± 1.93	33.88 ± 3.57	27.97 ± 2.59	34.53 ± 3.80
*t*	—	0.614	−5.402	0.082	−6.761
*P*	—	0.540	< 0.001	0.713	< 0.001

## Data Availability

The data used to support the findings of this study are available from the corresponding author upon request.
